The article "Nanoformulation of Tetrapyrroles Derivatives in Photodynamic Therapy: A Focus on Bacteriochlorin" was published in 2022. Journal: Evid Based Complement Alternat Med.

# Nanoformulation of Tetrapyrroles Derivatives in Photodynamic Therapy: A Focus on Bacteriochlorin

**DOI:** 10.1155/2022/3011918

**Published:** 2022-09-30

**Authors:** Pragya Pallavi, Karthick Harini, Vijaya Anand Arumugam, Pemula Gowtham, Koyeli Girigoswami, Saradhadevi Muthukrishnan, Agnishwar Girigoswami

**Affiliations:** ^1^Medical Bionanotechnology, Faculty of Allied Health Sciences, Chettinad Hospital & Research Institute (CHRI), Chettinad Academy of Research and Education (CARE), Kelambakkam, Chennai, TN 603103, India; ^2^Department of Human Genetics and Molecular Biology, Bharathiar University, Coimbatore, TN 641046, India; ^3^Department of Biochemistry, Bharathiar University, Coimbatore, TN 641046, India

## Abstract

Photodynamic therapy (PDT) is a well-known remedial treatment for cancer, infections, and various other diseases. PDT uses nontoxic dyes called photosensitizers (PS) that are activated in visible light at the proper wavelength to generate ROS (reactive oxygen species) that aid in killing tumor cells and destroying pathogenic microbes. Deciding a suitable photosensitizer is essential for enhancing the effectiveness of photodynamic therapy. It is challenging to choose the photosensitizer that is appropriate for specific pathological circumstances, such as different cancer species. Porphyrin, chlorin, and bacteriochlorin are tetrapyrroles used with proper functionalization in PDT, among which some compound has been clinically approved. Most photosensitizers are hydrophobic, have minimum solubility, and exhibit cytotoxicity due to the dispersion in biological fluid. This paper reviewed some nanotechnology-based strategies to overcome these drawbacks. In PDT, metal nanoparticles are widely used due to their enhanced surface plasmon resonance. The self-assembled nano-drug carriers like polymeric micelles, liposomes, and metal-based nanoparticles play a significant role in solubilizing the photosensitizer to make them biocompatible.

## 1. Introduction

Tetrapyrroles are a group of chemical compounds that have four pyrrole derivatives linked in a linear fashion or cyclic way through methine bridges [1]. Linear tetrapyrroles contain three methine bridges due to the cleavage of cyclic structures during their formation. The four pyrrole rings are denoted clockwise as A, B, C, and D in cyclic tetrapyrroles. The linear tetrapyrroles, when compared to cyclic tetrapyrroles, contain loosely bounded metals [2]. These macrocyclic compounds are widely found in nature to perform several biochemical functions in living organisms, like metabolism, transport of electrons, gases, and nutrients as part of the enzymes or proteins. Cyclic tetrapyrroles can easily form chelates with metal ions of iron, magnesium, cobalt, nickel, etc., to engage in biochemical functions that depend on their oxidation state and nature of chelated metal ions, including ring substituents, which can be used as effective photochemical reactants or catalysts [3, 4]. Tetrapyrroles with ring structures such as cobalt-containing substance-cobalamin are also known as corrinoids, which are distinguished by modifications in the fundamental porphyrin structure of chlorins, bacteriochlorins, porphyrin, heme *d*_1_, and siroheme (Figure 1) [5, 6]. The enzymes involved in the catalytic reaction of radical-based rearrangement utilize cobalamin as its cofactor. Chlorophyll *α* is a well-known chlorin-type molecule mostly found in green plants, cyanobacteria, and algae. Bacteriochlorophyll *α* is a part of the bacteriochlorin family and helps in the photosynthesis of some bacteria. On the opposite side of the macrocycle, bacteriochlorins have two reduced pyrroles, while chlorine has one reduced pyrrole, and porphyrin has a full tetrapyrrolic system [7]. Porphyrins are cyclic tetrapyrroles that play an important function in many biological processes. The heme is a porphyrin-based bioactive heterocyclic macromolecule compound present in hemoglobin [8]. It plays an important role as a cofactor in several enzymes like peroxidase, catalase, and cytochrome P-450. Cytochrome, which contains heme, is an essential component of several electron transport pathways. The iron in the heme fraction helps in respiration to transport carbon dioxide (CO_2_) and molecular oxygen (O_2_) through the circulatory system. Heme proteins can also be used as diatomic gas sensors for O_2_, CO_2_, and nitric oxide (NO) [9, 10].

The article "Nanoformulation of Tetrapyrroles Derivatives in Photodynamic Therapy: A Focus on Bacteriochlorin" was published in 2022. Journal: Evid Based Complement Alternat Med.

## 2. Biosynthetic Pathways of Tetrapyrroles

Tetrapyrroles are derived from a common precursor molecule, 5-aminolevulinic acid (ALA), via a biosynthetic pathway [11, 12]. The first step of conversion from 5-aminolevulinic acid (ALA) to uroporphyrinogen III occurs via enzymatic reaction. Uroporphyrinogen III is important to synthesize essential molecules such as heme, chlorophyll, vitamin B_12_, phytochromobilin, and coenzyme F_430_. The enzymes involved in the conversion of 5-aminolevulinic acid (ALA) to uroporphyrinogen III are uroporphyrinogen III synthase, porphobilinogen deaminase, and 5-aminolevulinic acid (ALA) dehydratase [13]. In the next step, uroporphyrinogen III gets converted to either precorrin 2 or coproporphyrinogen III. For the conversion of precorrin 2, the pathway involves the enzyme uroporphyrinogen III methyltransferase.

In order to synthesize chlorophyll and heme, uroporphyrinogen III undergoes a decarboxylation reaction with the enzyme called uroporphyrinogen III decarboxylase [14]. The tetrapyrrole biosynthetic pathway is elaborated as a schematic diagram in Figure 2. Ultimately, the end-products of the pathway vary in eukaryotes and prokaryotes according to the needs of the system.

The article "Nanoformulation of Tetrapyrroles Derivatives in Photodynamic Therapy: A Focus on Bacteriochlorin" was published in 2022. Journal: Evid Based Complement Alternat Med.

## 3. Classifications of Tetrapyrroles

Tetrapyrroles are classified into three broad groups—porphyrin, chlorin, and bacteriochlorin (Figure 3). A recent study showed the use of porphyrin, chlorin, and bacteriochlorin derivatives as photosensitizers (PS) due to their excellent physical properties, participation in the generation of high quantum yield, and absorption of light at certain higher wavelengths (600–750 nm) in the visible-NIR spectrum.

### 3.1. Porphyrins

Porphyrins have a well-balanced 18*π* aromatic macrocyclic structure that exists in all the living organisms on the Earth [15]. The methine group bridges the four pyrrole rings to shape porphyrin with an extended resonance structure. Protoporphyrin IX, including its iron derivatives heme and chlorophyll, is a remarkable example of natural porphyrins. Macrocyclic compounds like protoporphyrin IX (*λ*_max_ = 633 nm), chlorophyll-a (*λ*_max_ = 663 nm), and bacteriochlorophyll-1 (*λ*_max_ = 770 nm) absorb either at red or near-infrared (NIR) which is useful in light-driven photophysical processes. Dihydroporphyrins are the common form of reduced porphyrins, and the basic component of all these porphyrins is chlorin [16]. The 18 *π*-electrons out of 22 exist on the delocalization pathway to share these basic chromophoric structures. Due to their unique structure, porphyrins and metalloporphyrins can go for photoexcitation to generate reactive oxygen species [17]. Therefore, they are widely used as photosensitizers in photodynamic therapy.

Porphyrin derivatives are widely used in cancer therapy due to their strong absorption of light in the phototherapeutic region along with thermodynamically favorable photoinduced reaction with molecular oxygen to generate reactive oxygen species. The porphyrins possess good aromatic stability and can absorb visible or NIR radiation to generate a high amount of ROS. They have a structural diversity and can be functionalized very easily using simple chemical modifications. At the same time, their long triplet-state, half-life, and high ROS quantum yield with negligible dark toxicity made them ideal to be used as PS in photodynamic therapy. Hematoporphyrin derivatives and photofrins were the first generations of PS, showing higher uptake and good efficacy in the skin, brain, lung, and esophageal carcinomas [18]. Photofrin-driven PDT showed a commendable therapeutic effect against colorectal cancer, but their low light absorption became a challenge. Benzoporphyrins, phthalocyanines, purpurins, protoporphyrin IX, texaphyrins, and naphthalocyanine were the most popular second-generation PS [19]. Chemical modifications of second-generation PS are made for targeting accurately or, more specifically, generated 3^rd^ generation PS like mTHPC, chlorin e6, etc. [20]. The attachment of specific functional groups at the meso or beta position of the porphyrin ring created several new compounds for novel applications. Gomes et al. synthesized quinolones-linked porphyrins using Suzuki-Miyauracross-coupling reaction that showed high ROS production capacity for the treatment of leishmaniasis [21]. Abada et al. reported about the pyrrolidinone attached porphyrins for the assessment of antiparasitic activity [22]. Gomes et al., in 2015, reported that the metalloporphyrins coordinated with bismuth (III) and antimony (V), where antimony-coordinated metalloporphyrins had better ROS generation capacity and antiparasitic activity [23]. Das et al. reported that their synthesized porphyrin derivative 5,10-bis(4-carboxyphenyl)-15,20-bis(4-dimethylaminophenyl) has a catalytic inhibitory effect on the expression of human Top1 [24]. Presently, photosensitizers are being nanoformulated for better efficacy and increasing sensitivity in targeting diseased cells.

The article "Nanoformulation of Tetrapyrroles Derivatives in Photodynamic Therapy: A Focus on Bacteriochlorin" was published in 2022. Journal: Evid Based Complement Alternat Med.

### 3.2. Nanoformulated Porphyrins

Porphyrins and derivatives exhibit excellent photophysical, photochemical, and catalytic activity for the treatment of several diseases. However, the issues with photosensitizers like solubility, dark toxicity, and circulation half-life are the common reasons for their minimal efficacy [25, 26]. Nanotechnology offers certain possibilities to overcome challenges [27, 28]. In this regard, spherical vesicle-liposomes with an aqueous core surrounded by a lipid bilayer are well known to address biodistribution, bioavailability, biocompatibility, and cancer cell targeting [29–32]. Liposomes can transport the porphyrin of interest after solubilizing them to the diseased cells with a higher accumulation rate [33]. The solubility of hydrophobic porphyrin derivatives at the lipid bilayer of liposomes reduces the dark cytotoxicity. Dipalmitoylphosphatidylcholin (DPPC) liposomes were used to formulate zinc phthalocyanine for the enhancement of ROS quantum yield in the PDT against B16/F10 melanoma cells [34]. Hiraka et al. synthesized a pH-sensitive smart liposome combining cationic and anionic lipids with Fe-porphyrin to demonstrate the efficient PDT against MKN28 cell lines [35]. F127 polymer-based liposomes, in combination with graphene quantum dots and Zn-porphyrin, showed a synergistic effect of quantum dots and porphyrin on the ROS generation along with enhanced cellular uptake and stimuli-responsive drug release [36–38]. Kilian et al. reported porphyrin-phospholipid added liposomes for the light-triggered release of large biomolecules like dextran and fluorescent proteins [39]. Jiao et al. synthesized a porphyrin-based nano delivery system by iRGD-modified lipid-purpurin18 liposomes carrying sunitinib. The formulation offered synergistic treatment against the regression of tumors [40]. Cationic alkyl-porphyrins entrapped in POPC (palmitoyl-2-oleoyl-sn-glycero-3-phosphocholine) liposomes were reported by Giorgio et al. for the treatment of pancreatic cancer cells, which demonstrated a dual mechanism of cell death [39]. The applications of porphyrin-based liposomes are not limited to photodynamic therapy alone. It can carry the contrast agent or imaging agents along with the PS to provide the theranostic approaches [41].

The article "Nanoformulation of Tetrapyrroles Derivatives in Photodynamic Therapy: A Focus on Bacteriochlorin" was published in 2022. Journal: Evid Based Complement Alternat Med.

Like liposomes, dendrimers encapsulate functional materials like PS to improve the ROS quantum yield in PDT and targeted delivery. Generally, a convergent method is applied to synthesize the dendrimer-porphyrin and dendrimer-phthalocyanine to make them photo-functional nano-devices. Nishiyama et al. evaluated the efficacy of aryl ether dendrimer porphyrins. The formulation with 32 quaternary ammonium groups achieved remarkably higher ROS-induced toxicity to LLC cells than to 32 carboxylic groups containing supramolecular structures [42]. Militello et al. reported that the triplet state of meso-substituted tetraphenyl porphyrins at the PAMAM dendrimer branches facilitates an effective energy transfer to oxygen molecules to produce ROS that can be used in PDT [43]. Chung et al. synthesized a gold nanoshell coated with dendrimer porphyrin showing the synergistic effect of PDT and PTT (photothermal therapy) [44]. Rodriguez et al. used a 5-aminolevulinic acid dendrimer to synthesize the porphyrins for the treatment of cancer and atherosclerosis. They concluded that the 5-aminolevulinic acid dendrimer could be used in vascular PDT [45]. In the direction of improvement of therapeutic benefits and overcoming the fragile nature of liposomes, researchers developed cerasomes, which are hybrid nanoparticles composed of hydrophobic alkyl chains, hydrophilic lipids conjugated with triethoxysilane headgroups, and a connector group. Liang et al. prepared porphyrin-based cerasomes utilizing the sol-gel method. The synthesized formulations showed better stability and accumulation at the tumor site with improved bioavailability and ROS generation capacity upon irradiation of 400–700 nm light [46].

Penon et al. immobilized Zn-porphyrin derivative on the superparamagnetic iron oxide nanoparticles (SPION) to fabricate nanotools for PDT. The ROS production ability of the fabricated nanotools was better than the Zn-porphyrin derivative [47]. In 2017, Penon et al. synthesized AuNP conjugated with functionalized polyethylene glycol and alkanethiol (5-[4-(11-mercaptoundecyloxy)phenyl]-10,15,20-triphenylporphyrin, PR-SH) [48]. The AuNP produced by the monophasic method has the highest capacity to generate ROS than the biphasic one, which was used in the PDT test against cultured breast cancer cells SKBR-3. Zhang et al., in 2019, demonstrated the PDT and PTT simultaneously or synergistically functioned in a lung cancer model of the mouse with 660 and 808 nm laser irradiation after injecting 4-carboxyphenyl porphyrin conjugated gold nanorods coated silica. Porphyrin derivatives produced ROS for effective photodynamic therapy, and AuNP acted as a photothermal conversion agent [49]. Zeng et al. conducted a similar type of experiment utilizing AuNP after modifying with natural biopolymer chitosan using a ligand exchange method to enhance the stability and solubility of AuNP, reducing the overall cytotoxicity. The meso-tetrakis (4-sulphonatophenyl) porphyrin was then immobilized on the chitosan-encapsulated AuNPs for dual PTT and PDT. The formulated nanohybrids generated higher singlet oxygen than the porphyrin derivative alone and elevated the temperature up to 56°C, which was better than the bare AuNPs [50]. This is not all, but several pieces of research were recorded here to establish that the nanoformulated porphyrins are better in PDT compared to standard derivatives.

The article "Nanoformulation of Tetrapyrroles Derivatives in Photodynamic Therapy: A Focus on Bacteriochlorin" was published in 2022. Journal: Evid Based Complement Alternat Med.

## 4. Chlorin

The word chlorin is derived from chlorophyll, a photosynthetic pigment, the most prevalent source of chlorin [51]. The pigment resembles porphyrins structurally and has a magnesium ion at the core. The reduced chlorin variations are known as “bacteriochlorins” and “isobacteriochlorins” and are found in bacteriochlorophylls. Different synthetic chlorin analogs, including mono-L-aspartyl chlorin e6 and m-tetrahydroxyphenylchlorin (mTHPC), are useful as photosensitizers in photodynamic treatment [52]. Chlorophyll serves as an antioxidant that shields algal tissues from oxidative damage; in addition to its essential function in photosynthesis, it also acts as a protective factor against excessive UV radiation. Chlorin-based PS is getting a lot of attention compared to porphyrins because of their strong near-infrared absorption (>650 nm), which is relatively safe and penetrates deeply into biological tissues. Among them, temoporfin (m-THPC) and telaporfin (mono-L- aspartyl chlorin e6) were used for photodynamic treatment with additional benefits by enabling superficial impact and effective antimicrobial therapy [53].

The article "Nanoformulation of Tetrapyrroles Derivatives in Photodynamic Therapy: A Focus on Bacteriochlorin" was published in 2022. Journal: Evid Based Complement Alternat Med.

### 4.1. Nanoformulated Chlorin

Chlorins have high absorption in the red spectral region, making them a desirable substance for photodynamic treatment. Chlorin e6, the naturally occurring dye isolated from the plant during photosynthesis, is a derivative of chlorophylls [54]. The photosensitizer has a number of drawbacks, including poor solubility that can be the reason for aggregation, improper biodistribution, uncontrollable photo activity, and a slow rate of clearance, which can result in side effects after therapy. PDT using chlorin e6 is a very gentle technique with minimal to no adverse effects. PDT with chlorin e6 is usually sufficient in most situations. Photosensitizers have been used with nanoparticles or nanoscale drug delivery systems to increase the efficacy of treatment and minimize the drawbacks. Chang et al. studied two chlorin compounds, methyl pyropheophorbide-a (MPPa) and N-methoxyl purpurinimide (NMPi), as potential photosensitizers. The MPPa and NMPi show better results by the increase in phototoxicity *in vitro* depending on the concentration of PS, light irradiation, and changes in the volume and surface. The MPPa and NMPi can be promising PS for photodynamic activity both *in vivo* and *in vitro*. A significant contrast between their activity *in vivo* and the size of the initial tumor in mice was also observed, showing the need to treat cancer as early as possible [55]. Son et al. studied the conjugation of gelatin polymer with chlorin e6-2 and chlorin e6-8 to improve their solubility and ability for ROS generation. After the injection of gelatin-Ce6-2, it featured high accumulation in tumor tissue and prolonged blood circulation. This work reported that the PS in gelatin formulations has high solubility and stability. Gelatin enhanced the therapeutic effectiveness of Ce6 and superior tumor tissue accumulation during *in vivo* PDT [56]. Chitosan nanoparticle-loaded chlorin e6 (CNP-Ce6) was studied by Ding et al., and the result showed that in comparison to free Ce6, CNP-Ce6 enhanced the efficiency of PDT. This study using natural carriers provides a novel strategy to improve the therapeutic efficacy and biocompatibility of PDT [57]. Similarly, Yue et al. developed chitosan nanoformulations combined with photosensitizer Chlorin e6 in order to combat Gram-positive and Gram-negative bacteria. There were excellent ROS generation abilities and photodynamic antibacterial effects associated with the conjugates. There was a positive correlation between the degree of substitution and the formulations with chlorin e6 in the range of 4.81%–11.56%, which resulted in a stronger photodynamic antibacterial efficacy [58]. Amirshaghaghi et al. studied the chlorin e6 coated SPION nanoclusters (Ce6-SCs) synthesized by the oil-water emulsion method. The physicochemical properties of chlorin e6 can make hydrophobic SPION water-soluble nanoclusters without adding carriers or amphiphiles. Results showed that *in vivo* Ce6-SCs exhibit strong singlet oxygen production, significantly slowed tumor growth, and were accumulated in the tumor by enhanced permeability and retention [59]. Adimoolam et al. reported a study on chlorin e6 with lactoferrin nanoparticle, milk carrying iron Ce6-LfNPs and it showed that the production of ROS was increased in the formulations (Ce6-LfNPs) compared to free Ce6. Ce6-LfNPs were demonstrated to be nontoxic even if the concentration is ten times higher than that used in PDT. Ce6-LfNPs have potentiality in PDT by their high cellular uptake, efficient loading, and, more crucially, a huge decrease in IC_50_ values [60].

The article "Nanoformulation of Tetrapyrroles Derivatives in Photodynamic Therapy: A Focus on Bacteriochlorin" was published in 2022. Journal: Evid Based Complement Alternat Med.

## 5. Bacteriochlorins

Bacteriochlorins are composed of tetrapyrrole, where two pyrrole and two reduced pyrrole units are linked by methine linkages, with the two reduced pyrroles positioned diagonally across from one another. Bacteriochlorin is a class of hydroporphyrins that is porphyrin derivatives in which the addition of hydrogen or other substituents causes one or more double bonds to become saturated [61]. Nonmodified chlorophylls are too fragile for the majority of practical applications; however, some derivatives (such as Cu-chlorophyllin) are employed as the food and cosmetic colors as well as in photodynamic therapy in the treatment of tumors (chlorins and bacteriochlorins). For instance, the chlorophyll utilized in some health care products is a complicated combination of breakdown products [62]. Some photosynthetic bacteria can survive in the dark, producing bacteriochlorophyll *α*. However, the limitation in their uses makes it difficult to obtain other chlorophylls. Tetrahydroporphyrin-based compounds with a longer wavelength of absorption lying between 700 and 800 nm are now being developed as PS for PDT.

Numerous *de novo* synthetic approaches have been developed to obtain stable and efficient bacteriochlorins. Many of these methods generate bacteriochlorins with electron-withdrawing substituents. The stabilization of bacteriochlorin chromophore is due to geminal dimethyl groups and can be taken as an example [63]. As well as metal ions inserted into the macrocycle, exocyclic rings are present in the macrocycle, and halogen atoms are introduced in the meso-tetraphenyl bacteriochlorin to prevent oxidation. As a result of proper structural modifications to the macrocyclic ring, it has been possible to synthesize compounds with a wide range of substituents placed in various positions of the macrocyclic ring, allowing bacteriopyropheophorbides, and bacteriopurpurinimides, as well as tetraphenylbacteriochlorins to be obtained [64]. It is very important to note that metallo-bacteriochlorins are particularly significant for light harvesting and potential biomedical applications due to their strong NIR absorption. The use of metallo-bacteriochlorins, either standalone molecules or components of protein complexes, mimicking bacteriochlorophylls has been reported by many researchers.

The article "Nanoformulation of Tetrapyrroles Derivatives in Photodynamic Therapy: A Focus on Bacteriochlorin" was published in 2022. Journal: Evid Based Complement Alternat Med.

There is a central metal ion such as Mg^2+^ in both chlorophylls and bacteriochlorophylls [65]. Tetrapyrrole rings are known to change their electronic structure and photophysical properties when metals are inserted into them. There has been an increase in the absorption of the NIR that results from the progress of reducing the pyrrole rings. Bacteriochlorophylls a, b, and g absorb at 772 nm, 794 nm, and 762 nm, respectively, whereas chlorophyll a absorbs at 662 nm and 644 nm [66, 67]. A major limitation of bacteriochlorophylls is their instability and rigidity. The peripheral substitution of macrocycles, which affects their photophysical and spectroscopic properties, is an option for overcoming these limitations. This modification leads to an increase in low energy absorption bands towards the NIR wavelength while maintaining a constant energy level and lifetime of excited states, as well as an appropriate energy level for photochemical reactions to occur during the lifetime of these phases. Hence, semisynthetic or synthetic bacteriochlorins could be a good alternative to bacteriochlorophylls, becoming more attractive [64].

In order to synthesize compounds from bacteriochlorophylls, several divalent metallic ions, such as Zn^2+^, Cu^2+^, Co^2+^, and Pt^2+^, were coordinated using three main pathways. During the first step, a free macrocycle coordinates with Cd^2+^ before transmetalation [68, 69]. Additionally, Mg^2+^ was introduced via a Grignard reagent, and metal salts were directly reacted with. When metal ions are inserted into macrocycles, their electronic structure and optical properties are significantly altered. Porphyrins, whose symmetry rises from D2h to D4h, are particularly well described by structural changes. Depending on the type of metal ion, the Soret band may also undergo a bathochromic or hypsochromic shift. As a result of metal ion coordination, the low energy absorption band associated with the *S*_0_-*S*_1_ electronic transition undergoes a hypsochromic shift. The introduction of metal ions in the case of bacteriochlorins does not alter the symmetry of the structure at any time. However, it does cause a bathochromic shift at the band of absorption extending into the red part of the spectrum. Therefore, bacteriochlorophyll-a absorbs light at 772 nm while bacteriopheophytin-a absorbs light at 749 nm. In addition, it can be seen that metal insertion significantly increases the molar extinction coefficient [70].

The article "Nanoformulation of Tetrapyrroles Derivatives in Photodynamic Therapy: A Focus on Bacteriochlorin" was published in 2022. Journal: Evid Based Complement Alternat Med.

Photophysical and photochemical properties in bacteriopheophorbide can be affected by different types of metal ions. In diethyl ether, magnesium derivatives exhibit a fluorescence quantum yield equal to 0.1, a very long lifetime of the singlet excited state, and a relatively good quantum yield for intersystem crossing [71]. In comparison, the fluorescence quantum yield and the singlet excited state lifetime of zinc complexes are much lower. A heavy-atom effect can explain these differences, which are more pronounced in heavier metal complexes. When considering the influence of different metals on bacterial chlorophyll photophysical properties, it can be assumed that in nature, Mg^2+^ was selected over Zn^2+^ not only for its higher bioavailability but also for its ability to protect the photosynthetic machinery against excess ROS generation [72]. In contrast to magnesium-derived compounds, paramagnetic metal complexes with tetrapyrrolic ligands exhibit a more sophisticated effect. A high degree of internal conversion can be detected in such compounds, but no fluorescence can be observed. In addition, a paramagnetic metal ion is used by nature to prevent adverse photochemical reactions. In spite of the fact that these metalloporphyrins do not possess any photochemical activity, they are involved in significant redox reactions and therefore are associated with a wide range of biological processes [73].

### 5.1. The Basic Principle of Photodynamic Therapy

The term “photodynamic activity” is used to intensify the reactions occurring due to the exposure of light to a photo-sensitive material. This type of activity is used as a therapeutic strategy, mainly in the treatment of cancer, since the therapy can be performed highly localized. Recently, it has also been widely utilized to eliminate localized bacterial infections. The three components required to start a photochemical reaction are PS, a light source at visible or NIR, and oxygen molecules found in tissues [74]. These components work together to produce highly cytotoxic reactive oxygen species. Experiments conducted using PS for different types of diseases are tabulated in Table 1. After being injected, the photosensitizer is activated and goes through a number of photophysical and photochemical processes (Figure 4).

The article "Nanoformulation of Tetrapyrroles Derivatives in Photodynamic Therapy: A Focus on Bacteriochlorin" was published in 2022. Journal: Evid Based Complement Alternat Med.

The ROS is generated when photosensitizer in the excited state transmits an electron, a hydrogen atom, or energy to another molecule, such as O_2_. According to three linked anticancer processes, these species are implicated in the oxidative stress within the tumor by destroying biological structures. (i) indirect tumor blood vessel closure (ii) direct cytotoxic action leading to autophagy, necrosis, or apoptosis (cell self-healing process), and (iii) the production of proinflammatory processes, local and systemic immune system stimulation, and the eventual establishment of antitumor immunity. Each mechanism's contribution is influenced by the applied drug dosage, radiation dose, and interval between drug-to-light and level of oxygen in the cancerous site. The possibility of not only eliminating the main tumor but also avoiding metastases ultimately plays a significant role in the recovery from the disease and makes immune response against tumor tissues. Tetrapyrrolic macrocycles, such as bacteriochlorins and metallobacteriochlorins, are the most commonly used PDT photosensitizers. Clinically employed photosensitizers can either attach to plasma proteins (hydrophilic chemicals) or accumulate in various cellular compartments (higher lipophilic compounds), depending on their polarity. In addition, to create the best formulation and incubation period, the capacity of PS to accumulate in the tumor tissues and the intracellular localization should be identified, which also helps to identify the major site of photo-damage. The most significant toxic chemical in PDT is singlet oxygen, which causes photoinduced cellular damage.

### 5.2. Nanoformulated Bacteriochlorins

Many nanocarriers were developed to deliver the tetrapyrrole-based photosensitizer for drug delivery systems. Considering hydrophobicity, the major drawback of bacteriochlorophylls derivatives, Gomes et al. studied the bacteriochlorophylls *α* (Bchl *α*)-loaded poly (D, L-lactide-co-glycolide) nanoparticles synthesized using a solvent evaporation method. This method was mainly preferred for the encapsulation of Bchl *α*, and the experiments showed enhanced results due to the spectroscopic properties. Bchl *α* can be used as alternative molecules for PDT since they increase the generation of singlet oxygen. It was found that with this method, 69% of encapsulation was achieved. Based on the results of the spectroscopic analysis, the nanoparticles used as drug delivery systems show an absorption band drawn to the wavelength of 782 nm. Additionally, higher efficiency in singlet oxygen production was also observed, as well as a higher fluorescence quantum yield (*ΦF* = 0.19) [85]. Pantiushenko et al. synthesized a new type of material containing nonsulfur bacteriochlorophylls *α* and their derivatives. The photosensitizer N-aminobacteriopurpurinimide with lipoic acid moiety isolated from biomass of Rhodobacter capsulatus strain B10 nonsulfur purple bacterium. Lipoic acid is aurophilic because of its disulfide (S) moiety, which links gold (Au) nanoparticles through the S-Au bond. Due to nonspecific passive targeting, gold nanoparticles loaded with PS exhibit prolonged circulation time and improved tumor uptake compared to free photosensitizers [86]. Ostroverkhov et al. studied the immobilization of bacteriochlorin-based photosensitizer on magnetic nanoparticle (MNP) surface modified with human serum albumin MNP@PS. Despite being stable in water solution, MNP@PS complexes retained all of the photophysical properties of PS. There was a correlation between the length of the side chain, the size of MNP@PS, and the loading capacity of the cells. During the in vitro testing, MNP@PS was shown to be delivered to the cancer cells followed by a reaction resulting in photoinduced toxicity. MRI tracking of drug accumulation in tumors has been confirmed using as-synthesized complexes [87]. The new hybrid material is introduced by the metal-organic framework (MOFs) to avoid the disadvantage of traditional treatment. Zhang et al. prepared MOFs of bacteriochlorin-based photosensitizing agent absorbing in the NIR level for their application in photoacoustic imaging (PAI) guided photodynamic therapy. The hybrid nanomaterials are made of two major components—Hf_6_(_*μ*3_-O)_4_(_*μ*3_-OH)_4_ (DBBC-UiO) and H_2_DBBC (5,15-Di(p-benzoate) bacteriochlorin), where H_2_DBBC is present as a control cluster and also as blocks used for the treatment of hypoxic tumor because of its ability to generate ROS via photoreaction with singlet oxygen and hydroxyl radicals. This indicates DBBC-UiO MOF is oxygen-independent and used for effective therapy against hypoxic tumors, and it can be used as a diagnostic agent for cancer with deep penetration [88].

The article "Nanoformulation of Tetrapyrroles Derivatives in Photodynamic Therapy: A Focus on Bacteriochlorin" was published in 2022. Journal: Evid Based Complement Alternat Med.

## 6. Conclusion and Future Perspective

Photodynamic therapy is a multimodal diagnostic and therapeutic method with potential application in many fields. Photodynamic treatment is based on light and photosensitizing agents. PS agents are the natural structure that transmits light energy. PS absorbs visible light in a proper wavelength to generate ROS. The generated ROS helps to kill cancer cells and other pathogenic microbes. In this article, the specific physicochemical and spectroscopic characteristics of tetrapyrrolic photosensitizers are given a lot of attention. Nanoformulation of metal-based or polymer-based photosensitizers can actively reduce the detrimental effects of nude photosensitizers. Here, we can come to the conclusion that nanoformulated tetrapyrroles, especially bacteriochlorin, improve the therapeutic effect, including enhanced solubility, reducing dark toxicity, and regulating drug release. The use of photodynamic therapy with nanoformulation could revolutionize the field of theranostics for cancer and other infections.

There are several compounds that absorb NIR, but bacteriochlorins are particularly impressive. In various phototropic bacteria, there is a choice made by nature for them to conduct photosynthesis without the need for oxygen production. These molecules have been selected due to the fact that they are efficient at absorbing photons within a NIR range of 700–900 nm to have appropriate redox properties. It is most commonly known that bacteriochlorins are present in substances such as bacteriochlorophyll a, and stability is the main concern. It has become more and more important to obtain rationally designed or encapsulated synthetic bacteriochlorins in recent years, which can be used to obtain more favorable photochemical properties and increased stability. A wide range of practical applications was possible due to the introduction of various functional groups and metal ions into the bacterial chlorin core as well as the increased likelihood of obtaining large quantities of substantially pure metallobacteriochorins. Furthermore, it has been demonstrated that the functionalization of bacteriochlorins may enhance their effectiveness when encapsulated in polymeric micelles, nanoparticles, lipoproteins, and metal-organic frameworks. The combined effect of nanostructures on hybrid materials produces new interesting photochemical, photophysical, and redox properties that are not previously observed in these materials. Using the correct metals, ligands, supramolecular architecture, and anchored nanoparticles these essential properties of PS can be controlled in a smart manner. It is evident that nanoformulated derivatives are supporting the NIR region of the electromagnetic spectrum, a region that has never been used for so long at such a broad level.

## Figures and Tables

**Figure 1:** Structure of tetrapyrrole derivatives.

**Figure 2:** Synthesis pathway of tetrapyrroles.

**Figure 3:** Structure of classifications of tetrapyrrole.

**Figure 4:** Mechanism involved in photodynamic therapy.

**Table 1:** Research investigations with PDT for treating different types of disorders.

S.no	Photosensitizer	Study	Findings	Ref.
1.	5-ethylamino-9-diethylaminobenzo [a] phenothiazinium chloride (EtNBS)	Antimicrobial	(i) Two EtNBs derivatives were synthesized. (ii) Both were phototoxic to staphylococcus aureus 29213. (iii) But the carboxylic acid derivative was nontoxic to E. coli 25922.	[75]

2.	MB (methylene blue) with PLGA (polylactic-co-glycolic acid) (MBNP)	Antitumor	(i) Found that PLGA-coated MB inhibits the tumor growth (ii) Can be used in PDT and PTT-related anticancer therapies	[76]

3.	F, NCDs (fluorine and nitrogen co-doped carbon dot)	Antitumor	(i) F, NCDs exhibited a better effect on cell imaging and were a promising tool for hypoxia tumor microenvironment in PDT.	[77]

4.	Toluidine blue O (TBO) and radachlorin	Antimicrobial activity for dental caries and periodontal disease	(i) Found that Radachlorin® appears to be less effective than TBO-mediated photodynamic treatment at reducing streptococcus mutants *in vitro* viability.	[78]

5.	Six types of compound silicon and aluminum-based phthalocyanine	Cytotoxicity of V79 cell	(i) Found that compounds I and II have the same photocytotoxicity in comparison to AIPcOH.xH_2_O (ii) Compound IV showed more effective activity	[79]

6.	Indocynine green	Phototoxicity on normal cells-Skin fibroblast and human skin keratinocyte cells	(i) The concentration of photosensitizer affects the phototoxic effect on the cells. (ii) Photosensitizers in all tested concentrations damaged keratinocytes. (iii) Fibroblasts withstand only the energies of 4 and 10 g/mL of indocyanine green.	[80]

7.	Methylene blue	Anticancer- HT-29 cells (Colon)	(i) The mortality rate of the control group (A) and the treated group (B) were compared, and it was found that group B showed an 80% mortality rate.	[81]

8.	Diarylethene derivative DAE-TPE	Antitumor	(i) DAE-TPE NPs changed from their “opened” form (OF) to their “closed” form (CF) when exposed to UV light, which activated photosensitizer. (ii) The CF of DAE-TPE NPs were effective on cells	[82]

9.	Bacteriochlorin derivatives	Antitumor	(i) Due to their specific accumulation in tumor tissue and quick elimination from the body, photosensitizers (PS) demonstrated 100% tumor growth inhibition and 100% response rate in PDT.	[83]

10.	Photosensitizer encapsulated carbon dot (CQDs)	Antitumor-MCF-7 cells	(i) CQDs and HP-CQDs having high ROS generation properties in PDT cancer treatment	[84]

The article "Nanoformulation of Tetrapyrroles Derivatives in Photodynamic Therapy: A Focus on Bacteriochlorin" was published in 2022. Journal: Evid Based Complement Alternat Med.

## Data Availability

The authors confirm that the data supporting the findings of this study are available upon reasonable request with corresponding author.
